The article "Model of Urban Marketing Strategy Based on Ecological Environment Quality" was published in 2022. Journal: J Environ Public Health.

# Model of Urban Marketing Strategy Based on Ecological Environment Quality

**DOI:** 10.1155/2022/8096122

**Published:** 2022-08-08

**Authors:** Feihan Sun, Chongliang Ye, Weirong Zheng, Xumei Miao

**Affiliations:** ^1^Zhejiang College of Security Technology, Wenzhou 325016, China; ^2^Wenzhou Medical University, Wenzhou 325035, China; ^3^Shenzhen MSU-BIT University, Shenzhen 518172, China

## Abstract

Ecological environment quality is increasingly becoming a critical priority in measuring the sustainable development of modern cities. Reflecting on the reality of contemporary urban development, we create a structural equation model with city image and ecological quality as the antecedents of sustainable urban development, reflect on and expand the existing models of sustainable urban development, and further explore the mechanisms of various urban marketing factors on the shaping of city image. The study found that the continuous improvement of city marketing assets contributes to the process of shaping sustainable city branding. City image has a direct and significant positive impact on city recognition, city reputation, and perceived quality. Ecological environment quality also has a direct effect on city recognition and no direct effect on perceived quality or city reputation. However, ecological environment quality can affect city's reputation by acting on perceived quality through city recognition and then enhance the competitiveness of city sustainable development. The case practice of shaping a city's image by ecological environment quality illustrates the pragmatic return of humanism in contemporary urban development. While the halo effect of city image still exists, a good city reputation becomes another important influence on perceived quality and sustainability. This study facilitates the development of urban sustainable development theory and the extension of urban branding innovation theory, which will promote international dialogue in the field of urban eco-environment in China.

## 1. Introduction

The annual report on social mentality of China (2021) points out that in the process of social development toward common prosperity, the sense of ecological security is not advanced. Ecological environment quality is becoming a precious business card of city image, and an important assessment index for sustainable development of cities in postindustrial society, moreover, it is the way to green development of a region and a country [1]. City marketing based on ecological environment quality, as a distinction from the postindustrial city's economic development politics in response to the ecological environment impact of elite governance [2], more from the level of national marketing [3], to establish a sustainable development view of ecological and environmental policies affecting city image, driving the city faster, better and higher standards into the new vision of “Better City, Better Life” [4]. Urban marketing in postindustrial society is a process of innovative development and creative transformation of urban image, and it is also a contemporary interpretation of humanistic reversion, aiming at constructing a sustainable development paradigm with the integration of urban economic development, ecological environment, and cultural protection. Thus, the city's sustainable development competitiveness, green development index, city image, and quality of life can be significantly improved to realize the modernization of harmonious coexistence between humans and nature [5]. In addition, Sun and Ye [6] define city marketing as “the spatial expansion of social interactions with regional iconography.” This means that people's understanding of city image depends on their perceived socio-spatial relations, identity, and the differentiated connotation of city image in diverse geographical spaces, which provides the possibility of adding value to city image in a strategic sense by means of ecologically based city image in the cultural context of different target groups.

The article "Model of Urban Marketing Strategy Based on Ecological Environment Quality" was published in 2022. Journal: J Environ Public Health.

In parallel, with the advent of post-industrial society, knowledge economy, and creative era, spiritual production provides theoretical and practical paths to guide the sustainability of material production [7]. For local government, urban image production encompasses the preservation and transformation of built places, the creation of urban imagination and urban branding, and the reconstruction of social relations that people shape around the use of urban space. It is the interweaving and coexistence of three discourses: physical space transformation, spiritual space creation, and social space reconstruction [8]. The production of urban image is becoming increasingly common and ecological, and the needs of residents' life experiences are changing towards differentiation and complexity, but the desire for modern and better life is a significant development trend for the construction of urban image and self-enhancement [9]. However, distinct cities have remarkable variations in the level of productivity development, social governance, and quality of life, which achieve diverse ranges of urban experience creation in the synergetic creation of city marketing strategies and city images [10]. Unlike the city image constructed through the paths of tourism space [11], traditional cultural space [12], and new business consumption space [13], the city image shaping strategy targeting ecological environment quality responds to the needs of China entering a new stage of development in pursuit of high quality of life, and adapts to the identity reconstruction and expectations of local people for a new living environment.

The article "Model of Urban Marketing Strategy Based on Ecological Environment Quality" was published in 2022. Journal: J Environ Public Health.

In line with previous studies, the criteria for measuring the success of city marketing strategies are often based on the effective synergy of government publicity, media promotion, city industry construction, city operations, resource utilization, and event development [14]. Although studies have explored urban marketing and sustainable development, most are based on perspectives such as historical and cultural heritage [15], public policy [16], sporting events [17], marketing media [18], and an evaluation system of natural ecological environment quality by selecting indicators from air quality, greenness, resource consumption, and waste emissions [6, 19, 20]. Nevertheless, in the context of the constantly evolving international situation and the increasingly significant improvement of China's urban environment, it is worth further verifying and debating whether the existing theoretical models still have universal applicability and sufficient explanatory power. In postindustrial society, the pursuit of material satisfaction is far from satisfying human needs, and gaining spiritual satisfaction is often more likely to increase individual happiness and security, thus shaping people's new imagination of space to be able to establish a good image of space. Few studies have explored the human imagination of space and the construction of urban images from the perspective of focusing on the quality of natural ecological environment. Therefore, based on the background of “spatial imagination” and “humanistic turn,” the article further reflects on the contemporary urban development reality and verifies different influencing factors and mechanisms of urban marketing through empirical analysis of the case practice theoretical path of reshaping urban image by ecological environment quality. Meanwhile, it aims to expand the theoretical framework of sustainable urban development and provide case practice for contemporary urban ecology to fuel the value-added of urban image.

## 2. Literature Review and Research Hypothesis

Innovative development routes, the search for new economic driving points for cities, and a good image strategy for cities in parallel with economic transformation are paramount [21]. Cities with high recognition and reputation can gain a brand premium based on addressing audience needs [22]. The perceived quality of the city is exemplified by the audience getting spiritual pleasure and generating a sense of well-being and security to enhance the sustainable competitiveness of the city [23]. Stănciulescu [24] contends that the perceived quality of the city reveals the essence of city marketing and is the main source of realizing the value of the city's image. City reputation is also viewed by most scholars as the core of city marketing [25]. It is the basis for an assessment of the audience's experience of using urban space and the quality of services, indicating the city's own differentiated competitiveness, and is an important psychological consideration for the audience's final choice of consumption behavior, etc., [26]. In addition, it has also been noted that the value of a city's image is measured by the level of awareness it evokes in the audience, such as well-being [27]. The higher city recognition, the more information the audience is informed about the city and the more dominant the city is in the market [28]. Therefore, it is considered that city reputation, perceived quality, and city recognition are the three main dimensions of city marketing assets.

The article "Model of Urban Marketing Strategy Based on Ecological Environment Quality" was published in 2022. Journal: J Environ Public Health.

However, these 3 dimensions of city marketing assets are not irrelevant to each other. Zheng et al. [30] using community public sports services as a perspective, found that city recognition has a significant positive effect on city perceived quality, and city reputation is a mediating variable in the relationship between city recognition and city perceived quality. Molaei's [28] findings validated that both city recognition and city reputation have a significant effect on perceived quality. Du [29], after comparing the city marketing of Dalian, which enhances competitiveness with environment, and Qingdao, which strengthens industrialization, pointed out that there are significant differences between the city marketing of the two different development paths and that city recognition and city reputation directly or indirectly affect the perceived quality. Based on the abovementioned research insights, this paper proposes the following hypothesis.

 
*H*1: city recognition has a positive effect on perceived quality
 
*H*2: city reputation has a positive effect on perceived quality
 
*H*3: city recognition has a positive effect on city reputation

Well-being and security are the possibilities of the audience group's urban space utilization experience and service quality, and are the postpsychological stages of the audience group's spatial perception of the social development process [31]. Wang [21] stated that audience groups with high city marketing assets would respond more positively to city image shaping. Feihan et al. [7] posit that components of city marketing assets positively influence audience groups' perceptions and subsequent acquisition of a sense of urban well-being and security. Kim and Shim [32] conducted a study on the relationship and influence between spatial reputation and spatial well-being and security in a shopping place and showed that spatial reputation has a significant influence on spatial well-being and security. Zhang and Li [33] examined the well-being and security of tourist destinations and showed that perceived quality has a positive and significant effect on well-being and security. And Sun's [12] study on traditional cultural spaces in Suzhou showed that city recognition has a positive impact on well-being and security with perceived quality and city reputation as mediating variables and that when city recognition increases, perceived quality also increases and ultimately increases the competitiveness of the city for sustainable development. It can be seen that strengthening all dimensions of the city's marketing assets, it will help to form a good reputation and value for the city, establish positive experiences and values for the audience groups, and inspire a sense of well-being and security, thus forming a sustainable development of the city and the people's aspiration for a better life. Therefore, the following hypothesis is proposed:

 
*H*4: city recognition has a positive effect on well-being and security
 
*H*5: perceived quality has a positive effect on well-being and security
 
*H*6: city reputation has a positive effect on well-being and security

The concept of the urban image was initially proposed by Kevin Lynch [34] and refers to the ability of urban spaces to hold a public image among audience groups, consisting of five elements of a priori civic art traditions such as districts and landmarks, which in turn evoke mental images of audience groups, or Imageability [35]. Commonly, it is the description, word of mouth, or stereotype of a city, which is influenced by the quality of the city itself, its geographical features, economic and political background, and historical traditions [12]. Numerous audience groups tend to seek out city information to reduce the perceived risk of behavioral decisions before deciding where to work, where to live, or where to travel [36]. City image can be seen as a “guarantor” of a city's strategic positioning in the marketplace [37]. Dai and Zheng [38] revealed in their study of the city image of Nanjing, a historical and cultural city in China, that city image is a better predictor of audience groups' perceptions and evaluative attitudes toward the city. Audience groups prefer to associate products exported from areas with better image marketing compared to cities with positive evaluations of high quality, value, experience, and reliability [39]. This leads to the following hypothesis in this paper:

 
*H*7: city image has a positive effect on city recognition
 
*H*8: city image has a positive effect on perceived quality
 
*H*9: city image has a positive impact on city reputation

In an economy with an overproduction of commodities, ecological security is a materialistic act and a symbolic symbol that conveys people's quality of life, values, and cultural preferences [40]. In China, the pursuit of urban ecological environment quality has received unprecedented attention, and audience groups have begun to enjoy the pursuit of ecology, individuality, organic, sentiment and environmental protection, and actively advocate the pursuit of a high level of ecological quality that can satisfy physical and mental enjoyment and good living. As identification and symbolic marker of a consensus for a good life, the symbolic meaning and symbolic value implied by ecological environmental quality have also become the main purpose pursued by individuals. The important output form of Chinese ecologism is individual, scientific, systematic, strategic, historical, and global, and is a new banner for the construction of beautiful China [41]. The ecological environment quality concerning the good life becomes a capital that can be flaunted as a matter of an individual's spatial identity and taste, with symbolic socio-cultural significance [42]. As a derivative of post-industrial society, eco-environmental quality fully reflects people's human-oriented pursuit of environmental orientation, spatial imagination, cultural concept, and life experience is driven by modern governance, new media, and other technologies. Also, the pursuit of eco-environmental quality is not only at the city level but also at the individual level, and the cultural level has to be created collaboratively, which determines the need to realize individual perceptions, values, renewal, and leap forward of the city image through the added value of marketing [43]. Accordingly, the following hypothesis is formulated.

 
*H*10: ecological environment quality has a positive impact on city recognition
 
*H*11: ecological environment quality has a positive effect on perceived quality
 
*H*12: ecological environment quality has a positive effect on city reputation

Through the above literature review and research hypothesis, the following conceptual model is proposed to explore the path and factor analysis of urban marketing based on ecological environment quality (Figure 1).

The article "Model of Urban Marketing Strategy Based on Ecological Environment Quality" was published in 2022. Journal: J Environ Public Health.

## 3. Methodology

### 3.1. Case Descriptions

*W* city is located in the most developed Yangtze River Delta metropolitan area in China. In recent years, while economic strength has increased substantially, the system has advanced the reform of the ecological civilization system, and the construction of ecological civilization has become more effective, the quality of environmental beauty has become more distinct, and the people's sense of ecological well-being and security has been remarkably reinforced. The ecological and environmental development of *W* city has entered the strategic direction of carbon emission reduction, promoting pollution and carbon emission reduction synergy, promoting the comprehensive green transformation of economic and social development, and transforming ecological and environmental quality improvement from quantitative to qualitative [44].

In 2020, for instance, despite the impact of the epidemic, *W* City accomplished the action of zero direct discharge of sewage from 115 townships, 1,391 residential areas, and 63 industrial clusters, and fulfilled the technical transformation or new construction projects of 12 sewage plants with clean discharge. Ecological corridors are established in nature reserves, wetland parks, forest parks, etc., creating a greening rate of nearly 60% in the city. In addition, it also attaches importance to the conservation and management of biological species resources and the corresponding ecological security. Habitat improvement initiatives have solved problems such as environmental filth and disorder in rural areas, and have also boosted the civilization of the countryside. W city is a series of environmental management work, the initial realization of urban and rural ecological beauty of the whole area, and fully build into a beautiful China city model, the construction of a city suitable for living, entrepreneurship, and leisure [45]. Ecological environment quality is progressively becoming a salient factor in the behavioral decisions of audience groups and the experience of urban space in *W* city [46].

“Green water and green mountains are golden mountains” has become an important concept for the sustainable development of Chinese cities. Ecological environment quality has become a label for city image, high quality of life, etc. In the post-industrial society, talent has become the driving force of urban development, which can retain local people and also attract outsiders. *W* City, through marketing strategies, boosts the soft power of the city while building hard power, reinforces the well-being of its citizens, and makes ecological environment quality an important soft power for the city to attract talents. Marketing a favorable city image based on ecological environment quality makes green life a symbol of identity, interest, and taste for an individual in the city, and gradually evolves from a hard power of urban ecological construction to a “symbolic” soft power reflecting individuality and the pursuit of a good life [47]. According to the demographic data in the past five years, the population of *W* city is growing year by year, and it is among the top cities in the country in attracting talents to reside. It can be said that *W* city is a very representative typical case in the practice of city image sustainability upgrading, which has universal guiding significance for deepening the understanding of the ecological impact of nowadays globalization and the theory of innovative construction of city image in the Chinese economy and society.

The article "Model of Urban Marketing Strategy Based on Ecological Environment Quality" was published in 2022. Journal: J Environ Public Health.

### 3.2. Questionnaire Design and Variable Measurement

By tracking the results of the more recent literature, it was determined that the questionnaire contained six categories of city recognition, city reputation, perceived quality, well-being and security, city image, and ecological environment quality (Table 1), with a total of 27 questions, and the content of the questions was revised according to the actual case. The questionnaire was measured using a 5-point Likert scale, with higher scores indicating that the audience group agreed more vigorously with the description and, conversely, disagreed more heavily.

## 4. Result Analysis

### 4.1. Descriptive Statistical Analysis

Selected audience groups with a high perception of the city image of W as the research subjects, and official questionnaires were distributed through the (*Wenjuanxing*) website in February 2021. To ensure the quality of the online questionnaire, 20 questionnaires were first distributed for pre-study to adjust the questionnaire statements and estimate the questionnaire response time. The minimum required response time for the subjects was 1 min, and for the sake of prudence, any response time ≤1 min was considered invalid, and the maximum response time was not required. Finally, a total of 351 questionnaires were collected, 31 questionnaires with extreme values were excluded, and a total of 320 valid questionnaires were obtained, with an effective rate of 91.16%.

The demographic profile of the sample was as follows: 24% male and 76% female; approximately 79% of the study population was 18 to 36 years old. 83.9% of the respondents live in *W*, of which 66.3% are residents, 22.9% are newly settled citizens, and 10.8% are college students educated in *W* whose households are not in *W*. In terms of education level, 37.6% are graduates and above, 36.3% are bachelor's degrees, 15.7% are vocational college, and 10.4% are high school and below. The geographical distribution of the sample covers most provinces in China. Therefore, overall, the sample size of this study adequately includes audience groups of different geographic regions, different cultural levels, different age levels, and different origins in China, and the sample coverage and intra-group variability are high, which can ensure the reliability and generalizability of the analysis results.

The article "Model of Urban Marketing Strategy Based on Ecological Environment Quality" was published in 2022. Journal: J Environ Public Health.

The mean and standard deviation of each variable index were calculated using SPSS 19.0 software, and the results are shown in Table 2. The results show that the mean values of the samples are all >3, which is in the middle to the upper level, indicating that the audience groups generally have a positive attitude toward the measurement indicators. Among them, the mean value of each indicator of city image is >3.5, the mean value of each indicator of ecological environment quality is >3.2; the mean value of city recognition is >3.6, and the general mean value of city reputation is >3.1, while the mean value of perceived quality is >3.0, and the mean value of well-being and security is >3.0. The numerical interval of the standard deviation is (0.742, 1.011), indicating a low level of dispersion in the sample. The above comparative analysis of the mean values of each latent variable reveals that although the city image of *W* has established the recognition of eco-city through marketing strategies, the city reputation, perceived quality, and the sense of well-being and security of the audience groups are lower than the city image and positioning created by *W* itself.

### 4.2. Reliability and Validity

Exploratory factor analysis was performed on the data using SPSS 19.0 software, and the reliability of the variables was estimated using the internal consistency coefficient, Cronbach's *α*, in addition to the KMO test and Barlett's spherical test, and the results showed (Table 3) that the Cronbach's *α* values were all >0.77, indicating high reliability of the data. The factor loadings of each observation were >0.59, and the KMO values of the extracted common factors were ≥0.656, sig. <0.05, the Barlett's sphere tests were all significant, and the cumulative variance contributions were all over 64%, so the extracted six factors were reasonable [48]. The minimum Cronbach's *α* value for each latent variable was 0.773 > 0.7, indicating that the data had high reliability and internal consistency.

### 4.3. Validated Factor Analysis

The data validity mainly includes content validity, convergent validity, and discriminant validity. Content validity relies primarily on previous research scales and a combination of expert opinions to ensure this. Convergent and discriminant validity relied on validation factor analysis [48]. The great likelihood estimation procedure of Lisrel 8.72 software was used to perform validation factor analysis for the six concepts in the model, using the correlation coefficient matrix of each variable indicator as the input matrix. The results showed that *χ*^2^/df = 4.39 < 5; CFI = 0.96, NFI = 0.94, IFI = 0.96, RFI = 0.93, all >0.9; GFI = 0.73, slightly different from the general standard; RMSEM = 0.070 < 0.08, thus indicating a good fit of the econometric model to the data.

The article "Model of Urban Marketing Strategy Based on Ecological Environment Quality" was published in 2022. Journal: J Environ Public Health.

Convergent validity aims to measure the degree of association between different observed indicators under the same latent variable. If the factor loadings of the indicators in the econometric model are all highly significant, the data are considered to have good convergent validity. The results of the validated factor analysis of Lisrel 8.72 showed (Table 4) that the factor loadings of each indicator in the econometric model ranged from 0.60 to 0.89; the factor loadings of all indicators were significant (*T* ranged from 10.60 to 19.36), indicating a high convergent validity of each conceptual indicator.

Discriminant validity requires that the degree of association between different concepts is sufficiently low, and if the interval between the non-standardized solution and the standard error of plus or minus two times the correlation coefficient of each latent variable is calculated does not contain 1, then the validity of the data is good. The intervals formed by the non-standardized solution plus or minus two times the standard error of the correlation coefficients of each latent variable in this study all met the standard (Table 5).

### 4.4. Structural Equation Analysis of Conceptual Model

Structural equation analysis of the conceptual model was performed using the maximum likelihood estimation method of LISREL 8.72. After the initial run of data, the *t*-values of the paths between latent variables were obtained. Since the coefficients of the paths from “ecological environment quality to city reputation,” “city recognition to perceived quality,” and “ecological environment quality to perceived quality” are negative, and the ∣*T*∣ values of the two paths from “city reputation to well-being and security” and “city recognition to well-being and security” are <1.96, so they are all deleted. The best results obtained after necessary model corrections showed that except for AGFI = 0.68, RMR = 0.055, GFI = 0.73, and RMSEA = 0.12, which were slightly different from the general criteria, *χ*^2^/df = 4.38, NFI = 0.94, NNFI = 0.95, CFI = 0.96, IFI = 0.96, and RFI = 0.93 were all >0.90, all of which met the screening rules of the model indicators. With a sample size of <500 and a model that contains a large number of latent variables, it is difficult to fully achieve the generally determining fit, and only a majority of the indicators can be measured as closely as possible [49]. Therefore, the fit of the model to the data in this study can be considered good. The path depicted by the solid line in Figure 2 shows the role relationship between the variables. That is, city image directly affects city recognition, perceived quality, and city reputation, ecological environment quality directly affects city recognition and indirectly affects city reputation, and city recognition can only indirectly affect perceived quality and sense of well-being and security through city reputation.  Table 6 shows that *T*-values ranged from 2.32 to 11.88, preserving the path of significant standardized estimates of the relationship between variables.

The article "Model of Urban Marketing Strategy Based on Ecological Environment Quality" was published in 2022. Journal: J Environ Public Health.

Combining the results of the data in Tables 6 and 7 shows that city image and ecological environment quality have a positive and direct impact on city recognition, and further have an indirect positive impact on city reputation through city recognition. At the same time, city image also directly and positively affects the reputation and perceived quality of the city. In terms of the impact between city marketing asset dimensions and on well-being and security, city recognition has a significant positive impact on city reputation, city reputation has a significant positive impact on perceived quality, and perceived quality has a significant positive impact on well-being and security. The two hypotheses of “city recognition has a positive effect on perceived quality” and “city reputation has a positive effect on well-being and security” are not valid. This study does not support the 2 hypotheses, *H*11 and *H*12. And it is further found that the hypothesis of *H*4 is also not significant, i.e., not only does ecological environment quality have no significant effect on city reputation but also does not positively and significantly affect perceived quality. This suggests that in post-industrial society today, there is no once-and-for-all paradigm for the role of ecological environmental quality in influencing the process of city image construction. The preliminary analysis is because, with the economic development and the expansion of the international horizon, a good ecological environment quality has become a landscape that every city takes for granted, and thus does not directly shape the perceived quality as a result. The impact of city recognition on well-being and security is not significant because it only affects the audience's attention to the city and does not directly lead to well-being and security unless the audience goes through the process of experiencing the city. City recognition also does not necessarily contribute to perceived quality and a sense of well-being and security due to factors such as service quality, social governance, and consumption levels. Similarly, the perceived quality of a city does not directly lead to a sense of well-being and security but indirectly determines the behavioral decisions and psychological satisfaction of the audience only after various factors are combined to achieve a certain perceived quality. In addition, this study confirms the hypothesis that “city image has a positive effect on perceived quality (*H*8)” (Table 8).

The article "Model of Urban Marketing Strategy Based on Ecological Environment Quality" was published in 2022. Journal: J Environ Public Health.

## 5. Discussion and Conclusion

This paper develops a city marketing model based on ecological environment quality. City marketing promotes the self-expression and identification of the inner personality of the audience group, highlighting the characteristics of the difference in city image and discovering the core elements that distinguish city image from other cities will help the audience group to perceive the uniqueness, rarity, and authenticity of the city image, so that the audience group can gain a sense of well-being and security, etc. In postindustrial society, the audience group of *W* city does not passively receive city marketing messages, but reflects and shapes the meaning of city image through the perceived city qualities of ecological environment quality [6]. The multiple narratives produced by city images in social reality [50], along with globalization and the occurrence of audience perceptions, continue to innovate their distinctive personalities. Ecological environment quality provides precisely the necessary spatial hard and soft power base for understanding the meaning of urban marketing in various contexts.

The ecological environment quality has no direct impact on the reputation and perceived quality of the city, which is not in line with expectations. This paper postulates that with the development of the economy and the establishment of cultural confidence, nowadays people's ecological and environmental concepts are more rational and pragmatic. Second, globalization forces and local social development are interpenetrating and symbiotic, and the impact of globalization on ecological cities is a “localized” governance process [51], and improved ecological environments have become part of people's daily lifestyles. As urban development in China, today has popularized ecological environment construction, the extent to which urban ecological experience can directly meet the expectations of audience groups will determine whether they are willing to contribute to the sustainable development of the city. Therefore, this paper concludes that in the Chinese context of post-industrial social development, it is legitimate that there is no significant positive influence relationship between city reputation and perceived quality of audience groups based on the ecological environment of city image.

The article "Model of Urban Marketing Strategy Based on Ecological Environment Quality" was published in 2022. Journal: J Environ Public Health.

City reputation is an important mediator in shaping perceived quality, and perceived quality is the only path to a sense of well-being and security. City marketing needs to be based on strengthening the city's marketing assets [52]. From a marketing perspective, the higher the city's reputation, the better it is for the city to leverage the city's reputation to explore and address the lack of information in another emerging market in order to achieve city promotion goals across market segments. Compared with other city images, if the city's reputation is better, more stable, more innovative, and better able to enhance the quality and experience of the city, it will be more beneficial to enhance the perceived quality of the audience group in order to successfully implement the city marketing value. This study proves that only the advantage of having city recognition is far from enough. Perhaps the combination of ever-improving aesthetics, practicality that follows the development of modern technology, experience that surpasses psychological expectations, and accessibility to a high quality of life are the practical considerations that trigger the audience's current sense of well-being and security.

By conducting further discussions on two types of cultural geographic factors, such as city image effect and ecological environment quality, this paper proposes and empirically proves the path hypothesis of city marketing, enriches the case study object and is an expansion of city marketing theory. Theoretically, it will not only help to promote the theory of city brand marketing in terms of eco-environmental quality but also promote the international dialogue in the field of eco-environmental and sustainable urban development; practically, in future research, two types of cultural geographic factors, namely urban image effect and ecological quality, can be further studied and discussed in depth; also, the variation in city image evaluation and well-being and security of different audience groups can be further studied.

## Figures and Tables

**Figure 1:** Conceptual model of city marketing based on ecological environment quality.

**Figure 2:** Fitting effect of structural equation model.

The article "Model of Urban Marketing Strategy Based on Ecological Environment Quality" was published in 2022. Journal: J Environ Public Health.

**Table 1:** Conceptual index system.

Variable	Indicator
City recognition	CR1 *W* is a very well-known city in China
	CR2 Whenever eco-city is mentioned, one can think of *W*
	CR3 *W* is the best in eco-city

City reputation	CP1 A city of ecology, preferred *W*, surrounded by parks and green fields
	CP2 I can hear the insects and birds chirping.
	CP3 I don't want to leave *W*

Perceived quality	PQ1 *W*'s ecology is great
	PQ2 *W* has the best ecological environment among Chinese cities
	PQ3 *W* is trustworthy in ecological environment construction
	PQ4 I would recommend *W* to others

Well-being & security	WS1 I am willing to live in *W*
	WS2 I'll probably stay in *W*
	WS3 I always intend to develop in *W*
	WS4 I am extremely likely to choose *W* when working, traveling, etc.
	WS5 In order to settle in *W*, I will stay in *W* through employment, etc.

City image	CI1 Green shared city
	CI2 A city where people have a high quality of life
	CI3 Technologically advanced city
	CI4 A city with a high level of education
	CI5 Overall good feeling city
	CI6 City with less negative news
	CI7 A city with advanced ecological governance technology
	CI8 A city with sound ecological governance planning
	CI9 A city that has been successful in marketing eco-friendly concepts

Ecological quality	EQ1 A strong sense of personal satisfaction in living and working in a high-quality eco-friendly city
	EQ2 Having a good ecological environment makes me feel that the city is more civilized
	EQ3 Eco-friendly becomes a daily lifestyle routine for individuals

**Table 2:** Means and standard deviations of variables.

variable	Indicator	Mean	Standard deviation
City recognition	CRA	3.946	0.742
	CRB	3.611	0.958
City reputation	CPA	3.491	0.787
	CPB	3.101	0.860
Perceived quality	PQA	3.206	0.931
	PQB	3.051	1.011
Well-being & security	WSA	3.071	0.984
	WSB	3.501	0.891
City image	CIA	3.559	0.841
	CIB	3.574	0.851
Ecological quality	EQA	3.436	0.879
	EQB	3.251	0.915

*Note.* Each variable has two indicators, *A* and *B*. The relationship between each indicator and each scale in the questionnaire is as follows. Indicator value = Total score of items included in the indicator/number of items included in the indicator, e.g., CRA = (CR1 + CR3)/2.

**Table 3:** Data reliability.

Variable	Cronbach's *α*	KMO
City recognition	0.773	0.693
City reputation	0.821	0.714
Perceived quality	0.848	0.787
Well-being & security	0.858	0.818
City image	0.948	0.900
Ecological quality	0.805	0.656
Total	0.948	0.929

**Table 4:** Factor loadings and significant levels of indicators.

Variable	Indicator	Factor loading	*T* value
City recognition	CR1	0.69	11.21
	CR2	0.75	11.17
	CR3	0.82	11.92

City reputation	CP1	0.82	14.54
	CP2	0.81	14.85
	CP3	0.75	13.59

Perceived quality	PQ1	0.68	11.66
	PQ2	0.75	11.61
	PQ3	0.85	12.86
	PQ4	0.84	12.75

Well-being & security	WS1	0.80	15.28
	WS2	0.60	10.64
	WS3	0.85	16.33
	WS4	0.71	12.91
	WS5	0.78	14.70

City image	CI1	0.77	15.49
	CI2	0.77	15.74
	CI3	0.80	16.54
	CI4	0.85	18.09
	CI5	0.78	15.91
	CI6	0.81	16.94
	CI7	0.88	19.27
	CI8	0.88	19.12
	CI9	0.89	19.36

Ecological quality	EQ1	0.86	17.02
	EQ2	0.85	16.58
	EQ3	0.60	10.60

The article "Model of Urban Marketing Strategy Based on Ecological Environment Quality" was published in 2022. Journal: J Environ Public Health.

**Table 5:** Correlation coefficient and standard error of each latent variable.

	City image	Ecological quality	City recognition	City reputation	Perceived quality
Ecological quality	0.60 (0.05)				
City recognition	0.53 (0.09)	0.19 (0.08)			
City reputation	0.58 (0.08)	0.15 (0.07)	0.77 (0.10)		
Perceived quality	0.33 (0.05)	0.06 (0.03)	0.30 (0.06)	0.39 (0.06)	
Well-being & security	0.48 (0.07)	0.09 (0.04)	0.43 (0.08)	0.56 (0.08)	0.68 (0.13)

*Note.* The numbers outside the parentheses are the unstandardized values of the correlation coefficients, and the numbers inside the parentheses are the magnitude of the standard errors.

**Table 6:** Standardized estimates.

No.	Inter-variable relationship	Route	Standardized estimate	*T* value
1	City image⟶City recognition	*H*7	0.53	6.60
2	City image⟶City reputation	*H*9	0.18	2.57
3	City image⟶Perceived quality	*H*8	0.17	2.32
4	Ecological quality⟶City recognition	*H*10	0.19	2.50
5	City recognition⟶City reputation	*H*3	0.76	8.49
6	City reputation⟶Perceived quality	*H*2	0.60	7.04
7	Perceived quality⟶Well-being & security	*H*5	0.98	11.88

**Table 7:** Indirect effects between latent variables in the structural model.

	City image	Ecological quality	City recognition	City reputation
City reputation	0.08 (5.71)	0.07 (2.47)		
Perceived quality	0.05 (5.52)	0.03 (2.37)	0.06 (5.94)	
Well-being & security	0.07 (7.62)	0.04 (2.38)	0.08 (6.16)	0.08 (7.40)

*Note.* The number outside the parentheses indicates the standardized coefficient of indirect effects, and the number inside the parentheses indicates the *T*-value of this standardized coefficient.

**Table 8:** Hypothesis results.

Hypothesis	Result
*H*1: City recognition has a positive effect on perceived quality.	N
*H*2: City reputation has a positive effect on perceived quality.	Y
*H*3: City recognition has a positive effect on city reputation.	Y
*H*4: City recognition has a positive effect on well-being and security.	N
*H*5: Perceived quality has a positive effect on well-being and security.	Y
*H*6: City reputation has a positive effect on well-being and security.	N
*H*7: City image has a positive effect on city recognition.	Y
*H*8: City image has a positive effect on perceived quality.	Y
*H*9: City image has a positive impact on city reputation.	Y
*H*10: Ecological quality has a positive impact on city recognition.	Y
*H*11: Ecological quality has a positive effect on perceived quality.	N
*H*12: Ecological quality has a positive effect on city reputation.	N

The article "Model of Urban Marketing Strategy Based on Ecological Environment Quality" was published in 2022. Journal: J Environ Public Health.

## Data Availability

The data that support the findings of this study are available from the corresponding author upon reasonable request.
